# Organizational Silence among Hospital Nurses in China: A Cross-Sectional Study

This article has been retracted.

**DOI:** 10.1155/2022/9138644

**Published:** 2022-05-12

**Authors:** Jing Yang, Hui Yang, Binquan Wang

**Affiliations:** ^1^Nursing College, Shanxi Medical University, Taiyuan, Shanxi, China; ^2^First Hospital of Shanxi Medical University, Taiyuan, Shanxi, China

## Abstract

**Objective:**

To analyze the factors that contribute to organizational silence among Chinese nurses.

**Methods:**

A descriptive, comparative, and cross-sectional study was performed with the participation of 866 nurses from public hospitals in China. The data were collected using an online questionnaire that included sociodemographic information and a silence scale.

**Results:**

The overall level of organizational silence among nurses was moderate (51.35 ± 14.99). Nurses indicated that they remained silent about administrative (2.97 ± 1.10) and organizational topics (2.94 ± 1.11) yet were more vocal about matters related to responsibility (1.68 ± 0.86), honor (1.87 ± 0.95), and enthusiasm (2.07 ± 0.99). Moreover, data analysis demonstrated that department, educational status, professional title, years of employment, and employment status had effects on nurses' organizational silence (*p* < .05).

**Conclusion:**

This study provides information that could facilitate an understanding of organizational silence for both nurses and nursing managers. The results helped to identify the urgent need to adopt effective strategies to address the problem of nurses' organizational silence. Changes in management practices and organizational culture should be implemented to remove communication and other barriers that impede nurses' contributions to their organizations.

## 1. Introduction

The ability to address changes in a complex medical environment represents a constant challenge for organizations devoted to meeting the growing demand for health care services. Managers alone cannot resolve all the problems that arise. The rational allocation of human resources is a strategic factor to ensure the change and development of organizations [1]. Employee voice plays a crucial role in the smooth progress of that process, not only to deal with changes but also to achieve high-quality services [1, 2]. Nurses on the front line frequently are in a better position than their leaders to identify appropriate responses when problems exist or arise in the facilities where they work [3]. Unfortunately, nurses often choose not to share their views or make suggestions for a variety of reasons. Organizational silence occurs when most employees choose to remain silent [4]. A variety of stakeholders and scholars have come to recognize the importance of communication in healthcare settings. Research has illuminated the negative impact of organizational silence on efforts to promote personal growth and healthcare services [5–10]. However, there has been little research on organizational silence and nurses. This study addresses this gap in the literature by focusing specifically on nurses, employee voice, and silence. The study was designed to provide concrete suggestions for management practices that may reduce organizational silence among nurses.

Research on organizational silence emerged in the early 1960s. Scholars have developed a variety of approaches to the subject ever since. Rosen and Tesser found that employees were unwilling to convey harmful information to their leaders because they feared negative outcomes. They referred to this as the “mum effect,” and it continues to be an important management problem for public health and services. Organizational silence was first defined by Morrison and Milliken [4] as an employee's decision to remain silent with regard to their ideas, opinions, and suggestions on potential issues in the organization. Pinder and Harlos [11] defined organizational silence as an absence of voice; employees say or do very little about organizational issues in response to injustice and unfairness. Dyne et al. [12] noted that organizational silence was a multidimensional structure comprised of acquiescent silence, defensive silence, and prosocial silence. Xiaotao et al. (2008) described organizational silence as that which occurs when employees might have valuable perspectives based on their knowledge and direct experience about ways to improve their work or the workplace but refrain from sharing their opinions or suggestions.

Sharing information and knowledge proves crucial in efforts to confront novel and existing challenges in health care environments. Consequently, there has been a growing interest in organizational silence as well as a number of studies that have identified the problem specifically among nurses. A survey conducted in a public hospital in Turkey indicated that 65.7% of the nurses remained silent about matters related to work or the workplace [1]. Another study from Jordan found that approximately 81% of employees in 58 health centers kept silent and did not participate in decision making [13]. A sample of 205 Chinese ICU nurses also revealed a moderate level of organizational silence [14].

Studies have shown that organizational silence affects patient safety as well as individual and organizational development because of the lack of employee input about organizational issues. Nurses' thoughts about the safety of patients could help to prevent patient accidents [15]. Attree [16] showed that nurses in closed medical institutions were more likely to keep silent on issues related to patient safety. Moreover, there has been evidence that organizational silence has negatively impacted performance and job satisfaction, resulting in increased cynicism and resignations [2, 5, 17]. Similarly, Gambarotto and Cammozzo [18] noted that nurses' inability to express their inner thoughts for a long time had adverse effects on their physical and mental health. Organizational silence also impaired the health-care institutions' ability to identify errors. The missed opportunities to learn from employees impeded improvements and innovation [19].

Although there have been efforts in the health care sector to focus on the importance of communication and the inclusion of different voices for effective decision-making and to defend organizational interests, some employees have faced significant challenges in their communication with senior-level managers [1]. Studies on nurses have served to identify a variety of factors responsible for nurses' organizational silence. Some studies have demonstrated that organizational silence is associated with manager characteristics, including behavioral integrity, authority, leadership, and negative reactions to critical feedback [5, 13, 19–22]. In the United States, Manapragada and Bruk-lee [23] confirmed the relationship between an unfair organizational culture and organizational silence among nurses. Similarly, Gkorezis et al. [6] observed that nurses who perceived that ostracism or neglect existed in their institution tended to remain silent. Work-family conflict, family support, and interpersonal relationships also influenced organizational silence among nurses [22, 24]. Additionally, demographic characteristics such as clinical experience and education level have been important factors that influence nurse silence [10, 25].

An examination of organizational silence among nurses will provide information for administrators to help prevent its occurrence, ensure patient safety, and promote individual and organizational development.

## 2. Methods

### 2.1. Design

A descriptive, comparative, and cross-sectional study was conducted.

### 2.2. Participants

In this study, convenient sampling was used to recruit nurses from across the nation. The inclusion criteria were as follows: [13] agreed to participate in the study; [16] possessed a license to practice as a registered nurse; and [5] had worked in a hospital for at least half a year. Nurses were excluded if they had chronic health issues or mental problems. The appropriate sample size was determined by use of the Raosoft calculator. The minimum number of nurses necessary was determined to be 377 for a 5% margin of error and a confidence level of 95%. In anticipation of a 20% attrition rate, the sample was increased to 453.

### 2.3. Materials

Data were collected with a self-report questionnaire that included two parts. The first part was comprised of questions related to demographic characteristics, such as age, gender, department, educational status, professional title, years of work, and personnel management. The second part was the organizational silence scale developed by Rao soft Jing Yang and Hui Yang in 2016. The scale consists of 20 items with the following 4 dimensions: negative silence, defensive silence, prosocial silence, and disregard silence. Responses were scored on a five-point Likert scale. The responses ranged from 1 (definitely disagree) to 5 (definitely agree). The higher the score, the more serious the silent behavior. The overall Cronbach's *α* coefficient was 0.918, and the Cronbach's *α* coefficient of dimensions was between and 0.791 and 0.857. The content validity index was between 0.87 and 1.00, and the S-CVI was 0.94. The scale is a valid and reliable tool that researchers in China have used previously to evaluate nurses' organizational silence.

### 2.4. Data Collection

The data were collected from October to November 2019. Nurses who were willing to participate completed the online questionnaire anonymously. The instructions stipulated that the participants should submit the questionnaires within one week after receiving them. The investigators trained in questionnaire administration verified all the collected data and excluded the missing values or univariate outliers for further data analysis.

### 2.5. Data Analysis

The research team used IBM SPSS Statistics version 22.0 for Mac to analyze the collected data. All the outcome variables are described using descriptive analysis. Frequency count and percentage are used to describe the demographic characteristics. Means and standard deviation were conducted to evaluate the organizational silence of the respondents. Independent sample *t*-test and one-way ANOVA tests were performed to examine the respondents' organizational silence by demographic characteristics. The threshold for statistical significance was a *p* value of <0.05.

### 2.6. Ethical Considerations

Only deidentified data were collected and were thus considered exempt from institutional review board approval. Moreover, all the respondents volunteered to participate and no risks or harm was associated with the study.

## 3. Results

### 3.1. Sample Characteristics

This study included a sample of 866 nurses with a participation rate of 93.42%. The vast majority of the respondents (96.2%) were female; only 3.8% were male. Most of the respondents (*n* = 502; 58%) were between 20 and 29 years of age. A little over one-third were between the ages of 30 and 39 (*n* = 311; 35.9%). A small percentage were between the ages of 40 and 49 (*n* = 42; 4.8%) and even fewer were over 50 years of age (*n* = 11; 1.3%). The participants worked in a variety of units: internal medicine (29.8%), surgery (21%), gynecology (4.6%), pediatrics (7.2%), emergency (8.1%), ICU (10.6%), operation (4.5%), and others (14.2%). More than half of the nurses held a bachelor's degree (66.1%), and approximately one-third held an associate's degree (29.9%). Only 3.2% of the nurses were postgraduates, and 0.8% indicated that they held secondary technical school certificates. The majority (47.7%) of the participants were senior nurses. Only 3.5% of them were professors. A little over one-third (36.3%) of the nurses had between one and five years of work experience. Another third of the nurses (33.9%) had six to ten years of work experience, 12.2% had 11–15 years, and 10.2% had over 15 years. The remaining 7.4% had less than 1 year of experience. Most participants (81.9%) worked under a contract system, and 18.1% were full-time employees at the facilities where they worked (Table 1).

### 3.2. Organizational Silence among Study Participants

As displayed in Table 2, the total score of organizational silence among nurses was 51.35 ± 14.99. The highest score for organizational silence among the four dimensions was for negative silence (16.19 ± 5.02), followed by defensive silence (15.57 ± 5.66), prosocial silence (11.33 ± 3.67), and disregard silence (8.26 ± 3.15).

### 3.3. Impact of Demographic Variables on Organizational Silence

No significant relationships were found between individual demographic characteristics and organizational silence. However, one-way ANOVA for different departments revealed a significant difference in the score on organizational silence. Further analysis served to discover that the nurses who worked in the ICU had a higher score than those who worked in internal medicine (Table 3), trauma, and other departments (*p* values were, respectively, 0.004, 0.037, and 0.003). A significant relationship was also found between educational status and organizational silence (*p* < 0.001); higher education levels corresponded to higher scores on organizational silence. Organizational silence scores also coincided with higher-paying job classifications (*p* < 0.001). The difference between nurse and senior nurse was *p* = 0.013, the difference between nurse and charge nurse was *p* < 0.001, and the difference between nurse and professor of nursing was *p* = 0.018. Moreover, there was a statistically significant relationship between clinical experience and organizational silence; nurses who worked less than one year had a lower score than those who had worked for more than one year (*p* values for the different categories of work experience were 0.005, 0.001, 0.015, and 0.012, respectively). Finally, nurses who were full-time employees exhibited higher scores than those who worked under a contract system (*p* = 0.043).

## 4. Discussion

The overall score for organizational silence proved to be higher than average. A “lack of self-confidence” was the reason most often given for organizational silence. A review of the literature on nurse silence demonstrated that low self-esteem and self-confidence could make nurses think that they were not able to deal with work-related issues or problems [26]. The nurses frequently offered several reasons for their responses in the defensive and prosocial silence categories: a reluctance to challenge authority, consideration for their leaders' feelings, and a fear of disturbing a harmonious organizational atmosphere. These findings are consistent with the findings from previous studies that emphasized the important role that administrative and organizational reasons play in nurses' organizational silence. Nurses felt uncomfortable, feared discipline, and tended to remain silent in the presence of senior management [5, 22]. The disregard silence scores indicated that employees were unwilling to speak up because of their low level of organizational commitment. In our study, this dimension had the lowest score. It could be that Chinese nurses' sense of responsibility would inhibit actions motivated by a lack of commitment. These results are different from the observations made by Yurdakul et al. [10], in that most of the nurses in Turkey remained silent about matters related to ethics and responsibilities.

A number of studies have shown that organizational silence has been common among nurses. Significant changes would be required to reduce its occurrence in medical facilities. This study helped to identify the demographic factors that influenced nurses' organizational silence: department, education level, professional title, clinical experience, and personnel management. Consequently, these factors should be taken into consideration to understand the organizational silence of nurses in China.

There were significant differences in organizational silence among the units where the nurses work. Ciris [25] arrived at a similar conclusion. Recent studies have revealed that cultural dysfunction, poor administrative leadership, and complicated interpersonal relationships impacted nurses' willingness to share their opinions ([19, 22]; and [24]). Our results also showed that ICU nurses scored higher on organizational silence. Complex work environments could represent a contributing factor to the problem. ICU nurses tend to have heavier workloads and frequent interactions with professionals from other units, which could make it difficult for them to freely express their opinions.

The results from this study suggested that the level of organizational silence increased with educational status. However, previous work has shown that high school graduates tended to remain silent more than undergraduates and postgraduates due to a fear that speaking out might damage relationships and leave them isolated from their coworkers [10]. One possible explanation for the difference among Chinese nurses could be that there would be an incentive for those with lower levels of education to express their opinions. These nurses typically have experienced greater job insecurity precisely because they have less education, professional knowledge, income, and opportunities for promotions. Therefore, it could be that they were more inclined to speak up as a means by which to seek recognition, increase their self-esteem, and attempt to secure opportunities for professional development.

It was also noted that professional titles could affect nurses' organizational silence. This finding differed from the work by Seren Harmanci et al. [24], which revealed that there was no significant difference between position and organizational silence (*p* > 0.05). A possible explanation for this study's results could be that nurses with higher professional titles preferred to focus on their work content and ignored the importance of communicating with managers or colleagues because they were afraid of negative outcomes. Further research should be conducted to explore the impact of positions on nurses' organizational silence.

Another important finding was that nurses with the experience of less than one year had the lowest level of organizational silence compared with those with more than one year. However, this is inconsistent with previous studies that indicated that junior nurses were more silent. A possible explanation could be that junior nurses were more enthusiastic during their early stages of nursing work. Therefore, they were more inclined to communicate with head or senior nurses about the problems encountered in their work environment and not remain silent. This study also revealed that nurses with six to ten years of clinical experience exhibited the highest level of organizational silence. Ciris's work (2018) confirmed that nurses with six to twelve years of clinical experience were more silent than others due to fears related to employment.

Moreover, there was a significant effect on nurses' organizational silence in terms of employment status. Contract nurses actively expressed their opinions because they were worried about the stability and permanence of their job and hoped to be recognized. However, nurses on the regular payroll enjoyed greater job security, which contributed to a high level of organizational silence in their nursing practice. Therefore, nursing administrators should take this into account and take actions to help prevent this situation.

All other comparisons for age and gender were not statistically significant in this study. A number of previous studies found that there was a significant association between nurses' age and organizational silence [1, 10, 21, 25]. For instance, Alheet [13] and Hall et al. [21] reported that the age group of under 25 was more likely to remain silent in the organization. Ciris [25] also revealed that nurses of different ages had different levels of organizational silence. Additionally, two studies demonstrated that women kept more silent than men due to “fear of being isolated” and “fear of destroying interpersonal relationships” [1, 24]. However, our study reaffirmed the argument put forth by Yurdakul et al., in that there was no significant gender difference with regard to organizational silence.

## 5. Conclusions

The study showed that there exists a moderate level of organizational silence among Chinese nurses. Department, educational status, professional title, years of employment, and personnel management all impacted organizational silence. This study is one of the first comprehensive investigations to provide an examination of organizational silence among nurses working in China. Although studies have explored organizational silence among nurses, few studies have focused on Chinese nurses. The study had several limitations that merit mention. First, the organizational silence scale has been successfully used in China but may not capture the experiences of nurses in other countries. Future research could focus on other regions. Second, this research was a cross-sectional study. A study that tracks nurses over time may provide a greater understanding of the processes by which nurses develop workplace behaviors that motivate them to share their thoughts or remain silent. Finally, the low percentage of male participants was not representative of the nurse population in China, where approximately 3.8% of nurses are men.

The fact that organizational silence among nurses is so prevalent worldwide suggests a need for comprehensive strategies designed to eliminate the organizational and communicative barriers that inhibit employee contributions that could improve the delivery of health care services.

Organizational silence represents an important challenge for medical institutions because it adversely impacts the development of both individuals and organizations. Administrators play an important role in dealing with this issue. Too often management fails to cultivate an environment of trust with nurses. Consequently, nurses do not feel empowered to share their observations or express their opinions. Nurse managers and leaders need to be aware of the influencing factors of organizational silence in order to implement policies that can address this problem. There are at least two steps that could be taken in this direction. First, managers should create an atmosphere of trust to ensure that nurses may freely express their ideas and opinions. Second, managers should take steps to ensure the inclusion of different voices in the organization. Nurses should be encouraged to participate in organizational decision-making in order to promote organizational innovation and development.

## Figures and Tables

**Table 1:** Nurse demographic characteristics.

Variables	(*n*)	(%)
Age (years)		
20–29	502	58
30–39	311	35.9
40–49	42	4.8
50 and above	11	1.3
Gender		
Female	833	96.2
Male	33	3.8
Department		
Internal medicine	258	29.8
Surgery	182	21
Gynecology	40	4.6
Department of Pediatrics	62	7.2
Emergency room	70	8.1
ICU	92	10.6
Operation	39	4.5
Other	123	14.2
Educational status		
Secondary technical certificate	7	0.8
Associate's degree	259	29.9
Bachelor's degree	572	66.1
Postgraduate	28	3.2
Professional title		
Nurse	230	26.6
Senior nurse	413	47.7
Nurse in charge	193	22.3
Professor of nursing	30	3.5
Years of employment		
<1	64	7.4
1–5	314	36.3
6–10	294	33.9
11–15	106	12.2
>15	88	10.2
Personnel management		
Employee	157	18.1
Contract	709	81.9

**Table 2:** Summary of scores on organizational silence.

Scale and dimensions	Minimum	Maximum	Mean	SD
Negative silence	6.00	30.00	16.19	5.02
Defensive silence	6.00	30.00	15.57	5.66
Prosocial silence	4.00	20.00	11.33	3.67
Disregard silence	4.00	20.00	8.26	3.15
Total score	20.00	100.00	51.35	14.99

**Table 3:** Association between participants' demographic characteristics and organizational silence.

	Negative silence			Defensive silence			Prosocial silence			Disregard silence			Total score		
	M	SD	*p*	M	SD	*p*	M	SD	*p*	M	SD	*p*	M	SD	*p*
Age (years)															
20–29	15.94	4.98	0.112	15.50	5.63	0.111	11.22	3.64	0.310	8.28	3.18	0.501	50.94	15.07	0.155
30–39	16.41	5.03		15.65	5.74		11.40	3.74		8.20	3.06		51.66	14.86	
40–49	16.93	5.53		14.83	5.53		11.57	3.63		8.10	3.58		51.43	15.52	
50 and above	18.91	2.95		19.45	4.39		13.18	2.56		9.64	2.62		61.18	10.51	
Gender															
Female	16.17	4.98	0.425	15.53	5.65	0.259	11.28	3.67	0.079	8.23	3.11	0.167	51.21	14.93	0.158
Male	16.88	5.82		16.67	5.97		12.42	3.46		9.00	4.01		54.97	16.31	
Department															
Internal department	15.88	4.81	0.156	15.05	5.49	0.017^#^	10.98	3.65	0.063	8.17	2.94	0.561	50.09	14.63	0.036^#^
Surgical department	16.18	4.83		15.79	5.44		11.56	3.40		8.31	3.13		51.84	14.00	
Department of gynecology	15.80	4.94		15.33	6.17		10.70	3.82		8.23	2.85		50.05	15.13	
Department of pediatrics	16.95	4.17		16.22	4.65		11.31	2.68		8.44	2.72		52.92	11.47	
Emergency department	17.06	5.54		16.91	6.04^a^		11.53	4.03		8.43	3.75		53.93	17.00	
ICU	17.17	5.42^a^		16.92	6.08^a,f^		12.41	4.13^a,c^		8.80	3.56		55.32	16.38^a^	
Operation	15.46	5.58		14.69	5.75^e^		11.18	3.50		8.03	3.12		49.36	14.70^f^	
Other	15.63	5.23^f^		14.62	5.85^e,f^		11.02	3.83^f^		7.84	3.20^f^		49.11	15.92^e,f^	
Educational status															
Secondary/technical certificate	13.86	3.24	<0.001^#^	12.29	3.86	<0.001^#^	10.71	4.31	0.006^#^	6.57	3.26	<0.001^#^	43.43	12.16	<0.001^#^
Associate's degree	15.15	4.94		14.29	5.53		10.71	3.69		7.66	3.07		47.81	14.84	
Bachelor's degree	16.60	4.99^b1^		16.06	5.64^b1^		11.56	3.66^b1^		8.4	3.11^b1^		52.66	14.79^a1,b1^	
Postgraduate	18.14	5.00^a1b1^		18.32	5.28^a1,b1,c1^		12.46	2.63^b1^		10.57	3.13^a1,b1,c1^		59.50	13.94^a1,b1^	
Professional title															
Nurse	15.05	4.86	<0.001^#^	14.59	5.72	0.013^#^	10.90	3.73	0.016^#^	7.94	3.21	0.315	48.49	15.24	<0.001^#^
Senior nurse	16.23	4.97^a2^		15.75	5.56^a2^		11.23	3.70		8.34	3.15		51.55	14.84^a2^	
Nurse in charge	17.25	4.96^a2^		16.25	5.63^a2^		11.84	3.43^a2^		8.37	2.96		53.72	14.33^a2^	
Professor of nursing	17.73	5.48^a2^		16.37	6.09		12.50	3.76^a2^		8.73	3.76		55.33	16.18^a2^	
Years of working															
<1	14.13	4.18	0.003^#^	14.05	5.516	0.201	9.81	3.61	0.014^#^	7.70	2.95	0.454	45.69	13.92	0.032^#^
1–5	15.91	4.91^a3^		15.65	5.59^a3^		11.48	3.66^a3^		8.37	3.19		51.40	15.03^a3^	
6–10	16.59	5.20^a3^		15.93	5.82^a3^		11.43	3.62^a3^		8.39	3.16		52.34	15.21^a3^	
11–15	16.75	4.79^a3^		15.39	5.38		11.22	3.67^a3^		8.09	3.08		51.44	14.22^a3^	
>15	16.74	5.24^a3^		15.48	5.77		11.65	3.69^a3^		8.02	3.18		51.89	15.19^a3^	
Personnel management															
On the regular payroll	16.95	4.80	0.037^#^	16.05	5.21	0.244	11.68	3.24	0.148	8.87	3.09	0.007^#^	53.54	13.78	0.043^#^
In contract system	16.03	5.05		15.47	5.76		11.25	3.75		8.12	3.15		50.87	15.21	

The differences according to department: ^a^internal department, ^b^surgical department, ^c^department of gynecology, ^d^department of pediatrics, ^e^emergency department, ^f^ICU, ^g^operation, and ^h^other. The differences according to level of education: ^a1^secondary technical certificate, ^b1^associate's degree, ^c1^bachelor's degree, and ^d1^postgraduate. The differences according to employment status: ^a2^nurse, ^b2^senior nurse, ^c2^nurse in charge, and ^d2^professor of nursing. The differences according to years of employment: ^a3^<1, ^b3^1–5, ^c3^6–10, ^d3^11–15, and ^e3^>15. ^∗^*p* values of Student's *t*-test; ^#^*p* values of one-way ANOVA.

## Data Availability

The data used to support the findings of this study are included within the article.
